The article "Targeting Oxidative Stress and Endothelial Dysfunction Using Tanshinone IIA for the Treatment of Tissue Inflammation and Fibrosis" was published in 2022. Journal: Oxid Med Cell Longev.

# Targeting Oxidative Stress and Endothelial Dysfunction Using Tanshinone IIA for the Treatment of Tissue Inflammation and Fibrosis

**DOI:** 10.1155/2022/2811789

**Published:** 2022-04-07

**Authors:** Tsuo-Cheng Lu, Yi-Hsiu Wu, Wei-Yu Chen, Yu-Chiang Hung

**Affiliations:** ^1^Department of Chinese Medicine, College of Medicine, Kaohsiung Chang Gung Memorial Hospital and Chang Gung University, Kaohsiung, Taiwan; ^2^Institute for Translational Research in Biomedicine, Kaohsiung Chang Gung Memorial Hospital, Kaohsiung, Taiwan; ^3^Department of Biochemistry and Molecular Biology, College of Medicine, National Cheng Kung University, Tainan, Taiwan

## Abstract

*Salvia miltiorrhiza* Burge (Danshen), a member of the Lamiaceae family, has been used in traditional Chinese medicine for many centuries as a valuable medicinal herb with antioxidative, anti-inflammatory, and antifibrotic potential. Several evidence-based reports have suggested that *Salvia miltiorrhiza* and its components prevent vascular diseases, including myocardial infarction, myocardial ischemia/reperfusion injury, arrhythmia, cardiac hypertrophy, and cardiac fibrosis. Tanshinone IIA (TanIIA), a lipophilic component of *Salvia miltiorrhiza*, has gained attention because of its possible preventive and curative activity against cardiovascular disorders. TanIIA, which possesses antioxidative, anti-inflammatory, and antifibrotic properties, could be a key component in the therapeutic potential of *Salvia miltiorrhiza*. Vascular diseases are often initiated by endothelial dysfunction, which is accompanied by vascular inflammation and fibrosis. In this review, we summarize how TanIIA suppresses tissue inflammation and fibrosis through signaling pathways such as PI3K/Akt/mTOR/eNOS, TGF-*β*1/Smad2/3, NF-*κ*B, JNK/SAPK (stress-activated protein kinase)/MAPK, and ERK/Nrf2 pathways. In brief, this review illustrates the therapeutic value of TanIIA in the alleviation of oxidative stress, inflammation, and fibrosis, which are critical components of cardiovascular disorders.

## 1. Introduction

*Salvia miltiorrhiza* Bunge, known as Danshen in Chinese, is a member of the Labiatae family. The dried root of the rhizome of *Salvia miltiorrhiza* Burge has been widely used in traditional medicine in China and other oriental regions, especially for treating cardiovascular diseases like coronary heart disease, myocardial infarction (MI), angina pectoris, and atherosclerosis [1–3]. The adverse effects of the therapeutic components are often mild [4, 5]. Although dried roots have been used as herbal medicine for more than a thousand years, the study of therapeutic content in the plant did not start until the early 20th century [1].

The article "Targeting Oxidative Stress and Endothelial Dysfunction Using Tanshinone IIA for the Treatment of Tissue Inflammation and Fibrosis" was published in 2022. Journal: Oxid Med Cell Longev.

Endothelial dysfunction describes a series of pathogenics promoting the development of hypertension and atherosclerosis, including oxidative stress, vascular endothelium injury, inflammation, and loss of smooth muscle elasticity [6, 7]. In hyperglycemic or diabetic conditions, mitochondria lose their functions and the electron transport chain is uncoupled, generating reactive oxygen species (ROS) [8]. ROS promote ER stress and mitochondrial alterations, causing apoptosis of endothelial cells. Additionally, ROS-injured endothelial cells generate less nitric oxide (NO) but more endothelin-1 (ET-1), promoting vasoconstriction [9, 10]. Notably, imbalanced proinflammatory mediators also induce leakage of endothelial walls and increase leukocyte adhesion [11].

Tanshinones are a group of nonpolar lipid-soluble components in *Salvia miltiorrhiza* extract, recognized for their therapeutic activity in the treatment and control of various diseases, including cardiovascular diseases, hepatitis, chronic kidney injury, and even dysmenorrhea [12]. TanIIA is the most well-studied and pharmacologically active compound among lipid-soluble tanshinones [2, 13]. TanIIA has been shown to control the symptoms of cardiovascular disease models such as neointima hyperplasia, atherosclerotic calcification, diet-induced atherosclerosis, and aortic aneurysm [2]. Furthermore, TanIIA controls the development of cardiovascular disorders through multiple mechanisms, including reduction of lipid oxidation and ROS generation, antiapoptosis, anti-inflammation, and antifibrosis. These pathophysiological mechanisms are closely related to endothelial dysfunction. Here, we aimed to summarize the current understanding of the pharmacological activities of TanIIA in cardiovascular diseases with a focus on the antioxidation, anti-inflammatory, and antifibrotic effects of TanIIA.

## 2. *Salvia miltiorrhiza* and Its Derivatives

### 2.1. Compounds Derived from *Salvia miltiorrhiza*

Although *Salvia miltiorrhiza* has a long history of application in traditional medicine, the search for possible pharmacological components began in the 1930s [1]. More than 200 compounds have been identified [2]. These derivatives can be mainly classified into two categories: water-soluble phenolic compounds (such as salvianolic acid A, salvianolic acid B, protocatechuic aldehyde, lithospermic acid, danshensu, caffeic acid, and rosmarinic acid) [14–16] and lipid-soluble compounds (such as tanshinone I, tanshinone IIA, tanshinone IIB, cryptotanshinone, and dihydrotanshinone I) (Figure 1) [1, 17, 18]. Water-soluble compounds, such as salvianolates, are widely used in the treatment of coronary heart disease [19, 20]. In contrast, lipid-soluble compounds such as tanshinones are more effective against cardiovascular diseases (CVDs) and cerebrovascular diseases, including atherosclerosis, myocardial infarction, and cardiac hypertrophy [13, 21]. These ingredients from *Salvia miltiorrhiza* were reported to have benefits in microcirculation and could increase blood flow, dilate coronary arteries, and prevent myocardial ischemia, atherosclerosis, calcification, and aortic aneurysm formation. Owing to their different chemical structures, their pharmacological activities, pharmacokinetics, and clinical applications are different. Among these active ingredients, tanshinones are one of the most well studied compounds [17]. In this review, we specifically focused on the lipid-soluble tanshinone, tanshinone IIA.

The article "Targeting Oxidative Stress and Endothelial Dysfunction Using Tanshinone IIA for the Treatment of Tissue Inflammation and Fibrosis" was published in 2022. Journal: Oxid Med Cell Longev.

### 2.2. The Tanshinones

Tanshinones are quinone diterpenes that were first isolated from *Salvia miltiorrhiza* roots by Nakao in 1930 [22], and more diterpene compounds have been separated and identified since then. Most of them are diterpene quinone compounds such as tanshinone I, tanshinone IIA, tanshinone IIB, and cryptotanshinone [23]. Tanshinones are synthesized from the five-carbon precursors, isopentenyl pyrophosphate (IPP) and dimethylallyl pyrophosphate (DMAPP), which are produced by the mevalonate (MVA) and the 2-C-methyl-D-erythritol 4-phosphate (MEP) pathways (Figure 2(a)) [24, 25]. TanIIA was discovered considered the main active lipophilic constituent of *Salvia miltiorrhiza* [14]. The core structure of tanshinones contains four rings, including naphthalene or tetrahydronaphthalene rings A and B, ortho- or para-naphthoquinone or lactone ring C, and a furan or dihydrofuran ring D [14]. TanIIA and cryptotanshinone, which contain an ortho-quinone C-ring, are the most intensively studied compounds. However, their yield from cultured roots is low, and biotechnological approaches are needed to increase their productivity [24, 26]. Another issue with TanIIA is its low water solubility. Sodium TanIIA sulfonate (STS) is a derivative of TanIIA with a sodium sulfonate addition to the dihydrofuran ring at the C-16 position and hence exhibits increased polarity and water solubility (Figure 2(b)) [27–29]. STS often serves as a substitute for TanIIA, and it has been utilized interchangeably in many previous studies [28–30]. Both TanIIA and STS have been widely used in preclinical studies because of their anti-inflammatory, antioxidative, and antifibrotic properties [31]. However, some studies have claimed that the modification of the molecular structure changes the chemical properties and bioactivity [32–35].

In detail, the metabolic reaction of TanIIA and STS is similar in rat bile except for the oxidation in side chain, which occurred in TanIIA but not STS [35]. STS suppresses atorvastatin-driven cerebral hemorrhage in zebrafish embryos but not TanIIA [32]. Human Purinergic Receptor P2X7 is blocked by STS but not TanIIA [36]. On the other hand, TanIIA inhibits the phosphorylation of Akt when used with anticancer drug epirubicin and increase the apoptosis of breast cancer cell line BT-20. Yet, STS failed to be uptaken by the BT-20 [34]. TanIIA boosts the excretion of anticoagulant warfarin by structural modification. However, STS elevates warfarin concentration by dissociation of albumin-warfarin complex [33].

The article "Targeting Oxidative Stress and Endothelial Dysfunction Using Tanshinone IIA for the Treatment of Tissue Inflammation and Fibrosis" was published in 2022. Journal: Oxid Med Cell Longev.

Notably, TanIIA and STS exhibit different pharmacokinetic patterns. For intravenous injection, TanIIA showed elimination half-life of 1.0 ± 0.7 hour at 20 mg/kg and 1.8 ± 0.6 hour at 60 mg/kg dosage in the serum of male Sprague–Dawley rats [37]. STS showed terminal half-life for about 21.6 ± 2.4 minutes at 50 mg/kg dosage in the serum of Kunming male mice [38]. It seems that STS may exhibit a shorter half-life in animals based on the results above. Yet, the animal models, dosage, and the sensitivity of detection affect the calculated half-life in each model. In one study, STS exhibits a “distribution half-life (*t*_1/2*β*_)” of 0.91 ± 0.21 hour but “elimination half-life” (*t*_1/2*γ*_) for 13.45 hours when 2 mg/kg of STS were injected into male Sprague–Dawley rats [39], while the other study claimed only 26.57 minutes of elimination half-life at the dosage of 6 mg/kg [40]. The extended elimination half-life is partly due to the sensitivity of liquid chromatography-electrospray ionization-tandem mass spectrometry. Above all, a parallel comparison between the pharmacokinetics of TanIIA and STS is required to ascertain the faster turnover of STS.

For the tissue distribution, both TanIIA and STS can both found in organs like the heart, liver, spleen, and lung. For intravenous injection, TanIIA tends to reside in the lung and liver and STS tend to distribute in the kidney and liver [37, 38]. Interestingly, oral gavage of TanIIA resulted in accumulation of the compound in the gastrointestinal tract, reflecting the poor bioavailability of TanIIA [37].

Despite there being differences in pharmacokinetics and some molecular activities, both TanIIA and STS suppress endothelial dysfunction, the focus in this review. In this review, we summarized the studies using STS and TanIIA in vitro and in vivo in order to further explore the functional properties of these compounds (Tables 1 and 2).

## 3. Oxidative Stress and Endothelial Dysfunction in Tissue Inflammation and Fibrosis

### 3.1. Oxidative Stress in Tissue Inflammation and Fibrosis

Reactive oxygen species (ROS) are essential components of metabolism, immune responses, and cell signaling. However, excessive ROS threatens the normal function of cells. For example, oxidative stress damages DNA and alters protein structure into misfolded forms, causing stress to the cells and leading to cell senescence, apoptosis, or even necrosis [41, 42]. In endothelial cells, the nicotinamide adenine dinucleotide phosphate (NADPH) oxidase system (NOX) is the major source of ROS production, determined by NOX4 RNA within the cells [43]. In addition to endothelial cells, other cell types such as fibroblasts and leukocytes also express NOXs [44]. Notably, other enzymes such as cyclooxygenases, cytochrome P450 enzymes, and lipoxygenases, as well as organelles such as the endoplasmic reticulum (ER) and peroxisomes, generate ROS [41, 43].

The article "Targeting Oxidative Stress and Endothelial Dysfunction Using Tanshinone IIA for the Treatment of Tissue Inflammation and Fibrosis" was published in 2022. Journal: Oxid Med Cell Longev.

NOX expression can be triggered by physical stimuli, such as shear stress, growth factors, cytokines, and metabolic factors such as hyperglycemia. Downstream metabolites include (1) ONOO^−^ free radicals from NO oxidation, (2) increased ICAM/VCAM expression, (3) increased intracellular Ca2+ levels activating the MAPK and Akt pathways, and (4) increased collagen disposition [44].

ROS promote vascular fibrosis through several mechanisms. In fibroblasts, NOX4 promotes survival but suppresses cell death in models such as hypoxia [44, 45]. Furthermore, ROS and its generators, such as H_2_O_2_ and xanthine oxidase, reduced the RNA level of procollagens but boosted MMP-2, MMP-9, MMP-13, and fibronectin in cardiac fibroblasts [46]. In endothelial cells, NOX2 promotes endothelial-mesenchymal transition in the heart interstitium, worsening cardiac fibrosis if NOX2 transgenic mice were treated with angiotensin II (AngII) [47]. Finally, the ROS-generating enzyme gp91phox boosts ET-1 expression in vascular fibroblasts under AngII stimuli [48], indicating the involvement of oxidative stress in endothelial dysfunction and fibroblast activation. Oxidative stress-mediated endothelial dysfunction has recently been linked to the pathogenesis of COVID-19 [49]. This may explain the cardiovascular complications of COVID-19, considering the role of ROS in immune responses and tissue inflammation [50].

### 3.2. Endothelial Dysfunction Promotes Chronic Inflammation and Tissue Fibrosis

Endothelial cells are critical regulators of vascular tension. Mechanistically, the endothelium releases vasoconstrictors such as endothelin-1 (ET-1) and vasodilators such as nitric oxide (NO) [7]. Endothelial dysfunction describes a series of imbalanced endothelial regulations concerning redox status, vascular contraction, inflammation, and coagulation, leading to reduced elasticity of blood vessels and enhanced development of vascular plaque [51].

The article "Targeting Oxidative Stress and Endothelial Dysfunction Using Tanshinone IIA for the Treatment of Tissue Inflammation and Fibrosis" was published in 2022. Journal: Oxid Med Cell Longev.

The endothelium of blood vessels plays a critical role in inflammatory responses. For example, NO suppresses ET-1 expression and TNF-driven NF-*κ*B activation in endothelial cells [52]. Endothelial cells regulate inflammation through several mechanisms. First, the transmigration of leukocytes requires cell–cell interactions between leukocytes and endothelial cells. ICAM-1 is induced on the endothelial surface and binds to integrins (such as CD11b, CD18, and LFA-1) on the surface of leukocytes upon challenge with inflammatory stimuli [53]. Furthermore, activated NF-*κ*B in endothelial cells upregulates VCAM-1, which binds to very late antigen-4 (VLA-4, composed of CD49d and CD29) to recruit leukocytes [54]. Mechanical shear stress also synergizes with inflammatory cytokines to boost E-selectin expression, increasing the affinity of neutrophils to cultured human umbilical vein endothelial cells (HUVECs) [55]. Second, endothelial cells express chemokines required for leukocyte recruitment [56]. A classic example is interleukin-8, which is expressed in endothelial cells cultured under plaque-forming physical conditions [57]. Targeting the dysregulation of endothelial inflammation may be a potential treatment strategy for tissue fibrosis [58].

Below, we summarize the mechanism of action of TanIIA in the regulation of endothelial dysfunction and its potential implications for treating tissue inflammation and fibrosis (Figure 3 and Tables 1 and 2).

## 4. Mechanism of Action of TanIIA in Tissue Inflammation and Fibrosis

### 4.1. Antioxidation

The antioxidative activity of *Salvia miltiorrhiza* is well documented in cardiovascular diseases and anticancer therapy [59, 60]. Previous studies have pointed out that TanIIA quenches ROS through several mechanisms. First, TanIIA suppresses lipid peroxidation and DNA damage in mitochondria in the liver and heart [61, 62]. Notably, TanIIA directly scavenges adriamycin semiquinone free radicals when treated in heart homogenates in vitro [62]. In mitochondria, TanIIA can accept one electron from NADH dehydrogenase in complex I, which can be transferred to oxygen molecules or cytochrome c [63]. TanIIA also triggers redox-sensitive ERK/Nrf2/HO1 and AMPK/ACC (acetyl-coenzyme A carboxylase)/CPT1 (carnitine palmitoyltransferase-1) pathways, governing cell signaling through modulation of redox equilibrium [64].

The antioxidative effect of TanIIA has therapeutic potential in diseases other than CVD. For example, TanIIA reduced oxidative stress in the serum of tumor-bearing mice by combining intermittent hypoxia. TanIIA promotes apoptosis of tumor cells, which may be related to the activation of Nrf2 [65]. Similar protective effects were also observed in mice with experimental pancreatitis [66]. TanIIA shared protective signaling with the ROS scavenger NAC [66]. TanIIA may also contribute to antioxidative activity through other routes. For example, TanIIA induces the cAMP pathway to boost the expression of cystathionine-lyase C (CSE), which synthesizes hydrogen sulfide (H2S) and promotes antioxidative activity in HUVECs [67]. Additionally, TanIIA induced the lncRNA AK003290 in primary myocardial tissue from I/R-injured mice. AK003290 sponges the miRNA miR-124-5p and suppresses proapoptotic proteins such as BAX and ROS in cardiomyocytes. However, how TanIIA boosts lncRNA and how lncRNA regulates ROS levels are still elusive [68]. Our recent study revealed that *Salvia miltiorrhiza* aqueous extract could alleviate ROS-dependent cell apoptosis in adriamycin-induced cardiomyopathy [69], which further supports the antioxidative activity.

The article "Targeting Oxidative Stress and Endothelial Dysfunction Using Tanshinone IIA for the Treatment of Tissue Inflammation and Fibrosis" was published in 2022. Journal: Oxid Med Cell Longev.

### 4.2. Anti-Inflammation

Tanshinones possess anti-inflammatory effects and ameliorate many diseases. For example, tanshinone I possesses potency similar to that of celecoxib to suppress IL-1*β*-driven chondrocyte apoptosis, inflammation, and extracellular matrix degradation in cellular models and protects against bone erosion in an osteoarthritis model [70]. TanIIA also ameliorates the invasiveness of RA fibroblast-like synoviocytes by suppressing the PI3K-Akt, MAPK, and HIF-1*α* signaling pathways, which are downstream of TNF-*α* [71].

TanIIA also suppresses inflammatory responses in blood vessels, which are known to exacerbate endothelial dysfunction, atherosclerotic plaque formation, and vascular injury. The NF-*κ*B pathway, a potent proinflammatory circuit, can be inhibited by TanIIA, leading to the reduction of inflammatory mediators such as MCP-1, TGF-*β*, and TNF-*α*. The suppression of these cytokines also reduced macrophage infiltration into the infarcted myocardium [72, 73]. NF-*κ*B blockade also prevents the adhesion of TNF-*α*-driven endothelial progenitor cells (EPCs) by lowering the expression of ICAM-1 and VCAM-1 on the cell surface [74]. In addition, the NLRP3 inflammasome releases mature IL-1*β* and IL-18 in response to oxidative stress and danger signals upon myocardial infarction [75]. TanIIA was shown to block the NLRP3 inflammasome in a canine myocardial infarction model by restoring JAK-STAT and insulin signaling in the heart [76]. Moreover, a recent study found that TanIIA skews macrophages toward the M2 phenotype in vitro, boosting markers such as Fizz-1, Arginase-1, and CD206. The M2 polarization effect may be exerted by inhibition of the TLR4-HMGB1/CEBP-*β* pathway and reduction of miR-155 [77]. TanIIA exerts anti-inflammatory activity by blocking NF-*κ*B and NLRP3 inflammasomes but restores other signaling pathways.

The article "Targeting Oxidative Stress and Endothelial Dysfunction Using Tanshinone IIA for the Treatment of Tissue Inflammation and Fibrosis" was published in 2022. Journal: Oxid Med Cell Longev.

### 4.3. Inhibition of Canonical TGF-*β*-Mediated Fibrotic Pathway

TGF-*β* binds to a heterodimeric receptor composed of TGF-*β*RI and TGF-*β*RII. Upon TGF-*β* activation, TGF-*β*RI is phosphorylated by the kinase activity of TGF-*β*RII, providing a docking site for Smad2/3. Smad2/3 is phosphorylated by TGF-*β*RI and then binds to the co-Smad-like Smad4, which forms a complex and then translocates into the nucleus [78]. Profibrotic genes are actively transcribed once the Smad complex interacts with the Smad-binding element [79]. The Smad2/3 complex induces Foxm1, which boosts the expression of Snail [80]. Snail, Twist, and Slug are key transcription factors that suppress endothelial markers but boost mesenchymal markers [81]. For example, Snail suppresses E-cadherin and occludin expression but elevates mesenchymal markers FSP-1 and *α*-SMA (alpha-smooth muscle actin) [82]. In contrast, there is also a regulatory pathway mediated by Smad7, which blocks signal transduction from TGF-*β*RI [78].

TanIIA controls fibrosis by interfering with the Smad-dependent TGF-*β* pathway. In rat cardiac fibroblasts, TanIIA inhibits the phosphorylation of Smad2/3, leading to the reduction of nuclear translocation of Smads and downregulated expression of fibronectin genes [83, 84]. Similar regulatory mechanisms have also been found in STS-treated human atrial fibroblasts. In detail, TanIIA reduced the protein expression level of fibroblastic markers such as *α*-SMA, collagen type I and III, periostin, and TGF-*β* but elevated matrix metalloproteinase-1 (MMP-1) in AngII-treated cardiac fibroblasts [85–87], suggesting that TanIIA suppresses cardiac fibrosis [27].

The suppressive effect of TanIIA on Smad phosphorylation may be Nrf2-dependent [88]. TanIIA also demonstrated protective effects in animal models through Smad regulation. For example, TanIIA also protects against cardiac hypertrophy in hypertensive rats by downregulating Smad3 but upregulating Smad7 [89]. TanIIA-containing “Shensong Yangxin Capsule” suppresses Smad3 phosphorylation but boosts Smad7 expression, reduces cardiac fibrosis, and partly rescues cardiac function in the diabetic rodent model [90]. Notably, the antifibrotic effect of TanIIA can be expanded to other models. Recently, TanIIA was found to ameliorate silica-induced pulmonary fibrosis through the removal of triggering of the Nrf2 pathway, dephosphorylation of Smad3, and elevation of Smad7 [91–93].

### 4.4. Inhibition of Noncanonical TGF-*β*-Mediated Pathways

In addition to Smad phosphorylation, TGF-*β* also transmits noncanonical signals through the phosphorylation of MAPK family members, PI3K, Rho A, Rac, c-Abl, and PKC. Downstream genes include Snail1, Snail 2, and Twist1 [79]. For example, TGF-*β*2 drives EndMT in human cutaneous microvascular endothelial cells via collaborating with the Smad, MEK, PI3K, and p38 MAPK signaling pathways [81]. JAK2 also promotes pulmonary vascular remodeling through Smad3 sensitization in idiopathic pulmonary fibrosis models [94].

The article "Targeting Oxidative Stress and Endothelial Dysfunction Using Tanshinone IIA for the Treatment of Tissue Inflammation and Fibrosis" was published in 2022. Journal: Oxid Med Cell Longev.

STS has been shown to inhibit AngII-induced cardiomyocyte hypertrophy and lower systolic blood pressure in cultured neonatal rat myocardial cells in vitro and in rats in vivo, mainly through the suppression of c-Fos, c-Jun, ERK, and MEK [95–98]. The antifibrotic activity of STS has been demonstrated to inhibit TGF-*β*1-activated human atrial fibroblast-to-myofibroblast differentiation by suppressing both phosphorylation of Smad3 and ERK1/2 [99], suggesting that the antifibrotic functions of STS are tightly linked to its antioxidant activity. Notably, the antifibrotic effect of TanIIA is not limited to the cardiovascular system. A review article has summarized the antifibrotic effects of TanIIA on organs such as the lungs, kidneys, uterus, peritoneum, and retina [31].

### 4.5. Notch Pathway

The Notch pathway is essential for the development of vascular smooth muscle [100] and cardiac valves [101] in the embryonic stage. There are five transmembrane ligands (Jagged (Jag) 1 and Jag2, and Dll (delta-like) 1, Dll3, and Dll4) and four Notch receptors (Notch-1, Notch-2, Notch-3, and Notch-4) expressed on the cell surface. Binding of the ligand and Notch receptor triggers cleavage of the extracellular domain by ADAM and release of the Notch intracellular domain (NICD) by gamma-secretase, respectively. When released from the plasma membrane, NICD translocates into the nucleus and binds to the CSL (CBF1/Su(H)/LAG1) complex and MAML (mastermind-like protein), promoting the transcription of downstream genes such as NF-*κ*B, Akt, and p21 [78, 102]. In a fully grown cardiovascular system, Notch may promote EndMT in cardiovascular ECs [103]. For example, Notch-1 activation by Jag-1 induces Ca2+-sensing receptor (CASR) expression in pulmonary arterial smooth muscle cells (PASMCs), sensitizing right ventricular myocardial fibrosis in hypoxia-driven pulmonary hypertension rodent models [104]. By using hESC-derived endothelial cells, high-density culture activates Notch by Dll4 and Jag-1 expressed in other cells, promoting EndMT markers such as SMA, while suppressing CD31 expression [105].

TanIIA is known to suppress tumor progression through activation of the Notch signal pathway [106]. At an in vitro dosage of 1–50 *μ*M, TanIIA limits the growth, migration, and invasion of astrocytoma cells. At the molecular level, TanIIA boosts the expression of Notch-1 and caspase-3/9 but reduces the phosphorylation of c-Myc, MMP-9, and Bcl2 [107]. In the gastric cancer cell line SGC7901, TanIIA limits tumor proliferation and migration through suppression of FOXM1, a transcription factor that governs cell fate and promotes tumor progression and metastasis in multiple cancers [108]. Moreover, TanIIA protects spinal cord endothelium stability in injury models. In detail, STS at 3–10 *μ*M was found to promote the survival of spinal cord endothelial cells (SCMEC) in an oxygen-glucose deprivation model by boosting Notch signaling. In this case, Notch upregulation decreases inflammatory cytokines such as IL-6, TNF, and IL-1*β* in SCMECs. In the murine spinal cord injury model, STS can (1) boost the expression of Notch, (2) rescue the microvessel, (3) maintain the blood-spinal cord barrier, and (4) protect the structural and functional integrity of the nervous system [109]. However, whether the TanIIA-driven activation of Notch is beneficial or harmful for cardiovascular disorders is still uncertain. Further investigation of the TanIIA-Notch-EndMT crosstalk is required.

The article "Targeting Oxidative Stress and Endothelial Dysfunction Using Tanshinone IIA for the Treatment of Tissue Inflammation and Fibrosis" was published in 2022. Journal: Oxid Med Cell Longev.

### 4.6. Wnt Pathway

There are more than 10 Wnt genes in mammals, which share a conserved feature: palmitoylation on their polypeptide chain [110]. The lipid moiety is critical for the binding of Wnt proteins to frizzled receptors, a group of seven transmembrane proteins that provide a cysteine-rich ligand-binding site [111]. Without the Wnt ligand, the key signaling protein *β*-catenin is constantly quenched by a destruction complex, comprising proteins such as disheveled and GSK-3*β*, and then subjected to proteasomal degradation. Upon Wnt signal activation, *β*-catenin accumulates and translocates into the nucleus [112]. In the nucleus, *β*-catenin binds to T cell factors (TCFs) to induce the transcription of genes such as Twist [103]. Wnt signaling is crucial in the heart development, such as Wnt-*β*-catenin signaling is crucial for heart cushion formation through EndMT activity [113]. Nevertheless, Wnt signaling may result in pathogenic fibrosis in the adult heart. Wnt activation favors EndMT in the heart, which may be the cause of cardiac fibrosis. For example, increased Wnt ligands were found in the injured murine heart after acute myocardial infarction. In addition, GSK-3 inhibition and LAD ligation boost the endothelial expression of *β*-catenin, TCFs, and SMA in vitro and in vivo, respectively [114]. In clinical settings, cardiac samples from patients with idiopathic dilated cardiomyopathy (DCM) exhibit higher levels of Wnt, *β*-catenin, and snail expressions than those from normal subjects. The results fit the elevation of fibrosis markers such as SMA and FSP-1 in DCM patients [115].

The article "Targeting Oxidative Stress and Endothelial Dysfunction Using Tanshinone IIA for the Treatment of Tissue Inflammation and Fibrosis" was published in 2022. Journal: Oxid Med Cell Longev.

The therapeutic potential of the TanIIA-Wnt axis can be found in skin transplantation and cancer studies. At a dosage of approximately 5 *μ*M, TanIIA ameliorates ischemic skin flap mice by inducing the expression of *β*-catenin and stem cell markers such as SOX2, Nanog, and OCT4 in epidermal cells [116]. Nevertheless, at a dosage of 20 *μ*M, STS inhibited the expression levels of COX-2, *β*-catenin, and VEGF, resulting in growth inhibition of HC8693 colon cancer cells [117]. The regulatory role of TanIIA in the Wnt pathway seems contradictory, and the dosage and cell type should be taken into account.

TanIIA exerts protective effects by boosting the Wnt pathway in endothelial cells. For example, STS (~10 *μ*M) rescues the expression of *β*-catenin and the phosphorylation of GSK-3*β* in high-glucose-treated HUVECs. In contrast, STS treatment reduced apoptosis and the expression of CXCL1 in HUVEC [118]. Further improvement of HUVEC survival, inflammatory suppression, and production of NO can be found when STS is combined with ghrelin [119]. However, the antifibrotic effect of TanIIA can be demonstrated in spontaneously hypertensive rats (SHRs) by inhibiting the Wnt signaling pathway [120]. Intraperitoneal injection of 1 or 10 mg/kg TanIIA reduced cardiac Wnt2, *β*-catenin, and WISP-1. In addition, TanIIA readily reduces hypertrophy and fibrosis of the heart, especially the left ventricle. At the molecular level, TanIIA reduced the mRNA levels of Col1a1 and Col3a1. Moreover, TanIIA reduced cardiac injury markers such as troponin, NOX4, and ADMA, but elevated cardioprotective NO and eNOS. Functionally, TanIIA controls systolic blood pressure in SHR animals, regardless of dosage [120]. Although TanIIA is effective in many cardiovascular disorder models, it may not exert a simple molecular action to raise or lower the activity of the Wnt pathway. The therapeutic effect of Wnt regulation may depend on the cell type and disease conditions.

### 4.7. ET-1 Pathway

Endothelin-1 (ET-1) is encoded by EDN1. Full-length preproendothelin-1 is processed by furin, chymase, and neprilysin cleavage, leaving a 21-amino-acid peptide. ET-1 is the most potent member of the three endothelins found in mammals, largely derived from vascular endothelial cells in all types of blood vessels, although other cells such as macrophages, enteric glial cells, and some neurons express ET-1 as well. In addition to a constant expression, ET-1 in endothelial cells can be further boosted by pathophysiological stimuli. After release from the endothelium, ET-1 largely binds to a GPCR named ETA, but less so to the other GPCRs, ETB [121, 122]. ETA activation results in vasoconstriction of smooth muscle cells, making ET-1 a major culprit in cardiovascular disorders. However, the autocrine action of ET1 binds to ETB on endothelial cells, leading to the induction of the vasodilator NO. This may serve as a feedback mechanism to reduce vasoconstriction [121, 122]. The downstream pathway of ET includes phosphatidylinositol-specific phospholipase C (PI-PLC), digesting PIP2 into IP3 and diacylglycerol (DAG). IP3 induces cytosolic Ca2+ and then cell contraction, and DAG activates protein kinase C (PKC) signaling. In addition, ET activates RTK like Ras, transmitting the signal through RAF/MEK/MAPK [123].

The article "Targeting Oxidative Stress and Endothelial Dysfunction Using Tanshinone IIA for the Treatment of Tissue Inflammation and Fibrosis" was published in 2022. Journal: Oxid Med Cell Longev.

TanIIA suppresses ET-1-driven endothelial dysfunction at both the cellular and organ levels. In endothelial cells, TanIIA inhibits the expression of ET-1 in HUVEC under cyclic strain [124]. In smooth muscle cells, TanIIA reduced smooth muscle proliferation by blocking the ET-1/PDK1/AKT pathway [125]. In addition, TanIIA reduced cardiac fibroblast expansion by inhibiting AngII-driven ERK phosphorylation [126]. In chronic intermittent hypoxia models, TanIIA reduces ET-1 and ETA expressions but elevates ETB expression in the heart and aorta, thereby controlling blood pressure and ameliorating apoptosis and fibrosis of myocardium and blood vessels [127, 128].

### 4.8. CAV-1 Pathway

Caveolin-1 (CAV-1) is essential for the formation of caveolae and secretion of substances in the apical direction of vesicles. CAV-1 oligomerizes and is coated onto the surface of invaginated membrane structures [129]. In the vascular endothelium, CAV-1 is required for the transportation of LDL from the lumen to the vessel walls, forming atherosclerotic plaques [130, 131]. Genetic ablation of CAV-1 results in several physiological alterations. First, the lack of CAV-1 increased NO release and desensitized AngII, ET-1, and PMA-driven vasoconstriction, providing insight into the role of CAV-1 in maintenance of vascular stress [132]. Moreover, CAV-1 siRNA suppressed lipid transcytosis through the epithelium and diminished VCAM-1 expression and phosphorylation of NF-*κ*B p65 [131]. CAV-1 and TGF-*β* crosstalk can be found in vascular smooth muscle cells (VSMCs). CAV-1 is phosphorylated by c-Src upon TGF-*β* stimulation. Y14-phosphorylated CAV-1 activates Rho-GTP/ROCK signaling, which inhibits PTEN and phosphatase PPM1A. As a result, Smad2/3 phosphorylation is maintained and PAI-1 expression is increased in atherosclerotic plaques [133].

The article "Targeting Oxidative Stress and Endothelial Dysfunction Using Tanshinone IIA for the Treatment of Tissue Inflammation and Fibrosis" was published in 2022. Journal: Oxid Med Cell Longev.

TanIIA is known to control the downstream TGF-*β* pathway. Whether TanIIA directly controls the activity of CAV-1 in endothelial cells or VSMCs remains unknown. A previous study suggested the role of TanIIA in CAV-1-related endocytosis. In neuron progenitor cell lines, CAV-1 is essential for the endocytosis of TanIIA, promoting its biological activity in boosting MAPK42/44 and CREB activities. Furthermore, the entry of TanIIA elevates the expression levels of brain-derived neurotrophic factor (BDNF) and nerve growth factor (NGF) in these cell lines and promotes neuronal differentiation [134].

### 4.9. Other Mechanisms

As a broad-spectrum therapeutic compound, TanIIA also protects cardiovascular function through other mechanisms. In the hearts of the canine MI model, TanIIA restored PPAR-alpha expression but limited lipid accumulation [76]. TanIIA was found to protect against myocardial injury through boosting the expression of Bim, CHOP, and PDCD4 proteins and maintaining the phosphorylation of Akt, thus preventing apoptosis of cardiac tissues [135, 136]. Moreover, TanIIA-loaded nanoparticle was found to penetrate the blood–brain barrier and demonstrated a preventive effect against cerebral ischemia/reperfusion injury in rat models [137]. TanIIA was also found to reduce the expression and membrane translocation of intracellular chloride channel 1 (CLIC1), which is known responding to cellular oxidative stress and induces the expression of inflammatory cytokines. Furthermore, TanIIA treatment attenuates inflammatory cytokine expression, cellular ROS levels, ICAM-1/VCAM-1 expression, and atherosclerotic plaque formation [138]. TanIIA has also been shown to regulate vascular fibrosis through KLF4, which suppresses vascular remodeling, and consequently attenuates vascular neointimal hyperplasia in left common carotid artery-ligated mice [139]. Finally, a meta-analysis focusing on *Salvia miltiorrhiza* for the treatment of coronary heart disease was conducted after integrating the protein–protein interaction data. Tanshinones are proposed to regulate blood circulation through guanylate cyclase soluble subunit alpha-1 and guanylate cyclase soluble subunit beta-1 [140], thus providing insights for future studies on the regulatory effects of TanIIA.

## 5. Our Perspective

Recently, the medicinal value of Tan IIA, especially water-soluble STS, has been intensively explored. Cardiovascular application of TanIIA in combination with classical treatments dominates recent clinical trials. TanIIA has been found to improve the prognosis of coronary artery diseases by reducing injury markers, such as cardiac troponin-I, and the incidence of major adverse cardiovascular events [141–143]. As TanIIA inhibits high-sensitivity C-reactive protein (hs-CRP) and cytokines, such as MCP-1, in the blood, the anti-inflammatory role of TanIIA should be a key factor in ameliorating disease progression [141]. TanIIA also promotes vascular elasticity. Sanghuang–Danshen, a mixture of drugs containing TanIIA, reduced blood pressure and arterial stiffness in healthy smokers [144]. A recent meta-analysis revealed that TanIIA reduces blood pressure in patients with hypertensive nephropathy and improves renal function due to cardiac-renal crosstalk [145]. As detailed in the previous sections, cell and animal studies suggest that the antioxidative, anti-inflammatory, and antifibrotic effects of TanIIA may be the major contributing factors to its protective effect. The better understanding on the mechanism of action of these pathways may lead to identification of novel applications of TanIIA.

The article "Targeting Oxidative Stress and Endothelial Dysfunction Using Tanshinone IIA for the Treatment of Tissue Inflammation and Fibrosis" was published in 2022. Journal: Oxid Med Cell Longev.

## 6. Conclusion

Taken together, TanIIA, which possesses multifaceted roles involving antioxidation, anti-inflammation, and antifibrosis, could be a key component of *Salvia miltiorrhiza* with substantial therapeutic potential for cardiovascular disorders (Tables 1 and 2). In this review, we have summarized how TanIIA mediates its therapeutic activities against cardiovascular disorders via the suppression of endothelial dysfunction, tissue inflammation, and fibrosis through multiple signaling pathways. An improved understanding of the action of TanIIA in the amelioration of endothelial cell dysfunction may help to shed light on the molecular mechanisms and clinical implications of TanIIA for treating cardiovascular diseases associated with endothelial dysfunction and fibrosis.

## Figures and Tables

**Figure 1:** Major lipophilic and hydrophilic components of *Salvia miltiorrhiza*, obtained after modification from [21].

**Figure 2:** Biogenesis of tanshinones and the synthesis of STS. (a) Biogenesis of tanshinones. Obtained from [24] and modified. (b) Structure of TanIIA and STS. Obtained after modification from [27].

**Figure 3:** Summarized mechanism of action of tanshinone IIA in the prevention of endothelial dysfunction. Arrows (→) indicate the route of signaling involved in endothelial dysfunction. Factors suppressed by TanIIA are linked with (─┤). Endothelial dysfunction is a combination of oxidative stress, inflammation, and fibrosis of vascular endothelium. Aside from the antioxidative activity, TanIIA inhibits inflammatory signaling like the TLR4-NF-*κ*B axis and the MAPK pathway. TanIIA also blocks profibrotic components like TGF-*β*R1 and AT1R and the Wnt, Notch, and ET-1 signaling pathways.

The article "Targeting Oxidative Stress and Endothelial Dysfunction Using Tanshinone IIA for the Treatment of Tissue Inflammation and Fibrosis" was published in 2022. Journal: Oxid Med Cell Longev.

**Table 1:** Summarized in vitro mechanism of action of tanshinone IIA and STS.

Biological activity	Cell type	Model	Drug used	Drug dose	Timing	Key regulated factors	Physiological effect	Ref.
Antioxidative	Neonatal cardiac myocytes	H_2_O_2_-driven oxidative stress	TanIIA	0.01-0.1 *μ*M	24 h prior to oxidative stimuli	Prohibitin (↓)	Attenuates cell death	[146]
	Adult cardiac myocytes	I/R model Hypoxia	TanIIA	0.5-5 *μ*M	2 h before hypoxia	lncRNA AK003290 (↑) miR-124-5p (↓)	Decreases apoptosis rate and ROS production through activation of lncRNA AK003290	[68]
	Human umbilical vein endothelial cells (HUVECs)	Acrolein-induced oxidative cell injury	TanIIA	10-40 *μ*g/mL	3-12 h	Cystathionine *γ*-Lyase (CSE) (↑) H2S (↑) cAMP signaling (↑)	Attenuates oxidative endothelial injury through H_2_S	[67]

Anti-inflammatory	Rheumatoid arthritis, fibroblast-like synoviocytes (RA-FLS)	TNF-*α* induction	TanIIA	2.5-20 *μ*M	8-48 h	IL-6, IL-8, IL-1*β*, TNF-*α* (↓) MMPs (↓) p-p38, p-JNK, p-AKT, p-NF-*κ*B p65 (↓)	Reduces the viability, migration, and invasion of RA-FLSs	[71]
	RAW264.7 macrophages	LPS induction	TanIIA	0.1-10 *μ*M	30 min prior to LPS treatments	TLR4, COX-2, IL-1*β*, TNF-*α* (↓)	Alters microRNA profiles and reduces proinflammatory gene expression	[72]
	Bone marrow-derived endothelial progenitor cells from rats	TNF-*α* induction	TanIIA	1-20 *μ*M	18 h prior to TNF-*α* stimulation	VCAM-1, ICAM-1 (↓) p-NF-*κ*B, p-I*κ*B (↓)	Inhibits the adhesion of endothelial progenitor cells	[74]
	RAW264.7 macrophages	LPS induction	TanIIA	0.1-10 *μ*M	24 h	TLR4, HMGB1, iNOS (↓) IL-1*β*, TNF-*α* (↓) Arg1, FIZZ1, CEBP (↑) IL-10 (↑)	Elongates RAW264.7 cells, reduces mitochondrial Ca^2+^ level, and promotes M2 phenotypes.	[77]

Antifibrotic	Neonatal cardiac fibroblasts	TGF-*β*1 stimulation	TanIIA	1-100 *μ*M	2 h prior to TGF*β*1 stimulation	Fibronectin (↓) p-SMAD2/3 (↓)	Blocks nuclear translocation of pSmad-2/3	[83]
	Rat cardiac fibroblasts	X-rays irradiation	STS	10 *μ*M	1 h prior to irradiation	GRP78, CHOP (↓) ROS, IGF-1, p-SMAD2/3, Collagen-1 (↓)	Reduces irradiation-driven ROS generation and ER stress	[147]
	Rat atrial fibroblasts	TGF-*β*1 stimulation	STS	3-30 *μ*M	30 min prior to TGF-*β*1 treatments	p-SMAD2/3, p-ERK1/2 (↓) Collagens, *α*-SMA (↓)	Reduces TGF-*β*1-induced fibrotic markers	[99]
	Rat cardiac fibroblasts	Ang II stimulation	STS	3-30 *μ*M	30 min prior to Ang II treatments	p47phox (↓) Col1 (↓) MMP-1 (↑)	Attenuates Ang II-induced collagen expression and ROS generation	[85]
	Rat cardiac fibroblasts	TGF-*β*1 stimulation	STS	10-100 *μ*M	Pretreat	p-SMAD3 (↓) SMAD7 (↑) CTGF, COLI, *α*-SMA, vimentin (↓)	Reduces TGF-*β*1-driven fibrotic markers	[84]
	Human astrocytoma U-87MG cells	None	TanIIA	1-50 *μ*M	24-96 h	Notch-1, Casp-3/9 (↑) p-Myc, p-MMP-9, p-Bcl2 (↓)	Reduces proliferation and migration, but promotes cell death	[107]
	HUVEC cells	Cyclic strain	TanIIA	1-10 *μ*M	Cotreatment	ET-1 (↓) eNOS (↑) ATF3 (↑)	Attenuates cyclic strain-induced ET-1 expression	[124]
	Mouse neural stem cells (C17.2), Rat pheochromocytoma cells (PC12), embryonic Corticalneural stem cells	None	TanIIA	0.01-3 *μ*M	1-7 d	BDNF, NGF, GAP-43 (↑) p-MAPK42/44, p-CREB (↑) CAV-1 (↑)	Promotes neural differentiation	[134]

The article "Targeting Oxidative Stress and Endothelial Dysfunction Using Tanshinone IIA for the Treatment of Tissue Inflammation and Fibrosis" was published in 2022. Journal: Oxid Med Cell Longev.

**Table 2:** Summarized in vivo mechanism of action of tanshinone IIA and STS.

Biological activity	Animal	Disease model	Drug used	Drug dose	Timing	Key regulated factors	Physiological effect	Ref.
Antioxidative	Male Sprague–Dawley rats	High cholesterol diet-driven atherosclerotic calcification	TanIIA	35-70 mg/kg, oral	12 weeks	Cu/Zn SOD (↑) LDL (↓) Superoxide anion (↓)	Reduces atherosclerotic calcification	[148]
	Male–Sprague Dawley rats	Two-kidney, two-clip (2K2C) hypertensive rats	TanIIA	35-70 mg/(kg·d), oral	6 weeks (starting from 4 weeks after surgery)	Superoxide (↓) NOX2, NOX4, p47phox (↓)	Reduces myocardial fibrosis, cardiac hypertrophy and dysfunction	[149]
	Male C57BL/6 mice	LPS-induced cardiac fibrosis	TanIIA	10 mg/(kg·d), i.p.	2 weeks	gp91phox (↓), p67phox (↓) Collagens (↓), MMP2/9 (↓) TIMP1/2 (↓)	Suppresses cardiac fibrosis	[150]
	Male Sprague–Dawley rats	Isoproterenol-induced myocardial infarction	STS	4-16 mg/kg, i.v.	7 d (prior to ISO injection)	p-ERK1/2 (↓) SOD, GSH, GPx (↑) Nrf2, HO-1 (↑) AMPK/CPT-1 (↓)	Maintains the levels of circulating lipids and stabilizes cardiac functions	[64]
	Male ICR mice	Acute pancreatitis (caerulein, taurocholate injection)	STS	25 mg/kg, i.p.	2 h prior to surgery	Nrf2 (↑)	Ameliorates acute pancreatitis	[66]
	Male C57BL/6 mice	Lewis lung carcinoma + intermittent hypoxia	STS	10 mg/(kg·d), i.p.	5 weeks (starting from 5-7 d After tumor implantation)	Nrf2 (↑) MDA, SOD (↓) NF-*κ*B (↓)	Reduces tumor size driven by intermittent hypoxia	[65]

Anti-inflammatory	Male C57BL/6 mice	Adjuvant-induced arthritis (AIA)	TanIIA	30 mg/(kg·d), intragastric	2-31 d After arthritis induction	IL-6, IL-17, TNF-*α* (↓)	Ameliorates arthritis severity in AIA models	[71]
	Male ApoE−/− mice	High-fat diet	TanIIA	10-90 mg/(kg·d), gavage	13-26 weeks	TLR4, MyD88, NF-*κ*B (↓) MCP-1, TNF-*α* (↓)	Reduces atherosclerosis severity, stabilizes plaque, and decreases the blood lipid levels	[73]
	Male beagle dogs	Occlusion of left anterior descending	STS	1.3-5.2 mg/kg, i.v.	15 min After occlusion	TXNIP (↓), NLRP3 inflammasome, IL-18 (↓), p-JAK2, p-STAT3 (↓) SOSC3 (↑), p-insulin receptor, p-AkT, p-ERK1/2 (↑), PPAR*α* (↑)	Reduces myocardial infarct size and attenuates inflammatory cells infiltration	[76]

Anti-fibrotic	Spontaneously hypertensive rats	None	TanIIA	1-10 mg/(kg·week), i.p.	From 21 weeks	cTn-I, ADMA, Col1a1, Col3a1 (↓), NOX4 (↓), eNOS, NO (↑), Cys-C/Wnt signaling (↓)	Reduces systolic blood pressure and cardiac fibrosis in spontaneously hypertensive rats	[120]

The article "Targeting Oxidative Stress and Endothelial Dysfunction Using Tanshinone IIA for the Treatment of Tissue Inflammation and Fibrosis" was published in 2022. Journal: Oxid Med Cell Longev.

## Data Availability

No data were used to support this study.

## Abbreviations

ACC: Acetyl-coenzyme A carboxylase
ADAM: A disintegrin and metalloproteinase
ADMA: Asymmetric dimethylarginine
Akt: Protein kinase B, AKT serine/threonine kinase
AMPK: AMP-activated protein kinase
AngII: Angiotensin II
ATF3: Activating transcription factor 3
Bcl2: B cell lymphoma 2
BDNF: Brain-derived neurotrophic factor
Bim: Bcl-2-like protein 11
cAMP: Cyclic AMP
CAV-1: Caveolin-1
CEBP-*β*: CCAAT/enhancer-binding protein beta
CHOP: C/EBP homologous protein
CLIC1: Intracellular chloride channel 1
c-Myc: Cellular Myc protooncogene
COVID-19: Coronavirus disease 2019
CPT1: Carnitine palmitoyltransferase-1
CSE: Cystathionine *γ*-lyase
CSL: CBF1/Su(H)/LAG1
cTn: Cardiac troponin
DAG: Diacylglycerol
DCM: Dilated cardiomyopathy
Dll: Delta-like
EndMT: Endothelial-to-mesenchymal transition
eNOS: Endothelial nitric oxide synthase
ER: Endoplasmic reticulum
ERK: Extracellular signal-regulated kinase
ET-1: Endothelin-1
ETA and ETB: Endothelin receptors, type-A and type-B
Fizz1: Resistin-like alpha
FOXM1: Forkhead box protein M1
FSP-1: Fibroblast-specific protein 1
GAP43: Growth-associated protein 43
GSH: Glutathione
GSK: Glycogen synthase kinase
GUCY1A1: Guanylate cyclase soluble subunit alpha-1
GUCY1B1: Guanylate cyclase soluble subunit beta-1
H_2_S: Hydrogen sulfide
hESCs: Human embryonic stem cells
HIF-1*α*: Hypoxia-inducible factor 1-alpha
HMGB: High-mobility group box
HO-1: Heme oxygenase-1
HUVECs: Human umbilical vein endothelial cell
ICAM: Intercellular adhesion molecule
IGF-1: Insulin-like growth factor-1
IL-8: Interleukin-8
JAK: Janus kinases
JNK: c-Jun N-terminal kinases
KLF4: Kruppel-like factor 4
LAD: Left anterior descending coronary artery
LDL: Low-density lipoprotein
LFA-1: Lymphocyte function-associated antigen 1, integrin, alpha L
lncRNA: Long noncoding RNA
MAML: Mastermind-like protein
MAPK: Mitogen-activated protein kinase
MCP-1: Monocyte chemoattractant protein-1, CCL2
MDA: 3,4-Methylenedioxyamphetamine
MEK: MAPK/ERK kinase
MI: Myocardial infarction
MMP: Matrix metalloproteinase
mTOR: Mammalian target of rapamycin
MyD88: Myeloid differentiation primary response 88
NADPH: Nicotinamide adenine dinucleotide phosphate
NF-*κ*B: Nuclear factor kappa B
NGF: Nerve growth factor
NICD: Notch intracellular domain
NLRP3: NOD-, LRR-, and pyrin domain-containing protein 3
NO: Nitric oxide
NOX: NADPH-oxidase
Nrf2: Nuclear factor erythroid 2-related factor 2
OCT4: Octamer-binding transcription factor 4
ONOO^−^: Nitrate free radical
PAI-1: Plasminogen activator inhibitor 1
PDCD4: Programmed cell death 4
PDK1: Phosphoinositide-dependent kinase-1
PI3K: Phosphoinositide 3-kinase
PI-PLC: Phosphatidylinositol-specific phospholipase C
PKC: Protein kinase C
PPAR: Peroxisome proliferator-activated receptor
PPM1A: Protein phosphatase, Mg^2+^/Mn^2+^-dependent 1A
PTEN: Phosphatase and tensin homolog
RAF: Rapidly accelerated fibrosarcoma
ROCK: Rho-associated protein kinase
ROS: Reactive oxygen species
SAPK: Stress-activated protein kinase
SMA: Smooth muscle actin
Smad: Mothers against decapentaplegic homolog
SOD: Superoxide dismutase
SOSC: Suppressor of cytokine signaling 1
SOX2: SRY- (sex determining region Y-) box 2
STAT: Signal transducer and activator of transcription proteins
STS: Sodium tanshinone IIA sulfonate
TanIIA: Tanshinone IIA
TCF: T cell factor
TGF-*β*: Transforming growth factor, beta
TIMP: Tissue inhibitor of metalloproteinases
TLR: Toll-like receptors
TNF: Tumor necrosis factor
TNXNIP: Thioredoxin-interacting protein
VCAM: Vascular cell adhesion protein
VLA: Very late antigen
VSMC: Vascular smooth muscle cell
WISP1: WNT1-inducible signaling pathway protein 1
Wnt: Wingless-related integration site
